The article "MiR-192-5p Alleviated Fibrosis and Inflammatory Responses of Tendon Cells by Targeting NFAT5" was retracted in 2023. Reasons: signs of a paper mill; suspected computer-generated content; unreliable results or conclusions; concerns about the data.

# MiR-192-5p Alleviated Fibrosis and Inflammatory Responses of Tendon Cells by Targeting NFAT5

**DOI:** 10.1155/2022/6481846

**Published:** 2022-07-05

**Authors:** Fan Gong, Xiaoliang Li, Hanling Zhang, Jianke Wu, Guoxu Ma, Bowen Zhang, Jian Gao, Yi Ding, Yonglu Huang, Kun Xia, Suoli Cheng, Xuebing Zhou, Jiandang Shi, Fei Zhao

**Affiliations:** Hand & foot & Reconstruction Microsurgery, People's Hospital of Ningxia Hui Autonomous Region (The First Affiliated Hospital of Northwest University for Nationalities), Yinchuan, 750002 Ningxia, China

## Abstract

**Objective:**

To explore the effect of microRNA (miR)-192-5p on the inflammatory and fibrotic responses of tendon cells.

**Methods:**

Tendon cells were treated with transforming growth factor-*β*1 (TGF-*β*1). The expression of miR-192-5p and nuclear factor of activated T cells 5 (NFAT5) in tendon cells were detected by RT-qPCR. The expressions of inflammatory and fibrosis-related factors were detected by RT-qPCR and Western blot. MiR-192-5p binds to NFAT5 targeting by TargetScan and dual-luciferase reporter gene assay. The expression of the NFAT5 gene was detected by RT-qPCR and Western blot. Detection of apoptosis in tendon cells by flow cytometry.

**Results:**

MiR-192-5p was downregulated in tendon cells, and the expression level gradually decreased with the prolong of TGF-*β*1 treatment. The expression of NFAT5 increased with the treatment time of TGF-*β*1. The expression of miR-192-5p decreased collagen III (COLIII), *α* smooth muscle actin (*α*-SMA), matrix metalloproteinase- (MMP-) 1, and MMP-8 expression, thereby inhibiting TGF-*β*1-induced fibrosis in tendon cells. The expression of miR-192-5p decreased the expression of tumor necrosis factor-*α* (TNF-*α*), interleukin (IL)-6, and IL-1*β*, thereby alleviating TGF-*β*1-induced inflammatory response and reduce apoptosis in tendon cells. NFAT5 is a direct target of miR-192-5p in tendon cells. The upregulation of NFAT5 reversed the effect of miR-192-5p on the fibrotic activity and inflammatory response of TGF-*β*1-stimulated tendon cells.

**Conclusions:**

MiR-192-5p alleviates fibrosis and inflammatory responses of tendon cells by targeting NFAT5.

## 1. Introduction

Tendons are a crucial component of the musculoskeletal system [1], and tendon injury is a common damage in patients of all ages [2]. Following injury, the tendon heals poorly through a slow process, forming fibrous scar tissue with low biomechanical function [3]. Fibrosis healing is an overgenerated extracellular matrix, which will lead to continuous scar formation, hinder the normal structure and function of the healing tissue, and eventually form fibrous adhesion between the tendon and the surrounding tissue [4, 5]. At present, the main treatment method for tendon fibrosis and adhesion is conservative treatment and functional exercise. For severe damage, surgery is needed to rebuild the tendon [6–8]. To explore better treatment methods, it is necessary to understand the occurrence and development of tendon fibrosis at the molecular level.

Tendon fibrosis is a complex process, but some studies on the role of microRNA (miRNA) in tendon fibrosis have good effects. Cui et al. found that bone marrow macrophages secreted exosomes of miR-21-5p, which directly targeted Smad7, thereby regulating the activation of tendon cells fiber formation [9]. At the same time, Chen et al. confirmed that chitosan can inhibit the growth of fibroblasts by controlling the overexpression of miR-29b, downregulating the level of transforming growth factor-*β*1 (TGF-*β*1)/Smad3, and thus play a preventive role on tendon adhesion in the process of tendon healing [10]. The above evidence suggests that microRNA may play a role in regulating the process of tendon fibrosis.

microRNA (miR)-192-5p is a conserved miRNA that is abundant in the liver [11]. Flammang et al. demonstrated that miR-192-5p has tumor-suppressive effects in pancreatic ductal adenocarcinoma and is a high-potential diagnostic and prognostic marker [12]. However, the most of the studies on miR-192-5p have focused on liver cancer [13], breast cancer [14], and lung cancer [15]. Zhang et al. showed that miR-192-5p overexpression could promote apoptosis in hepatocytes [16]. Tang et al. also found in their study that miR-192-5p could regulate apoptosis in cholangiocarcinoma cells [17]. In addition, it has been shown that miR-192-5p plays a key role in inflammation in nonalcoholic fatty liver disease [18]. Other studies have shown that overexpression of miR-192-5p promotes inflammatory responses in mice with Alzheimer's disease [19]. The current study also found that miR-192-5p also has a potential role in the pathogenesis of kidney tubulointerstitial fibrosis [20].

This study aimed to examine the effects of miR-192-5p on TGF-*β*1-stimulated tendon cells' fibrosis and inflammation. The above studies have shown that miR-192-5p plays a role in apoptosis, inflammation, and fibrosis. However, its presence in tendon has been rarely studied. To explore the potential role of miR-192-5p in tendon fibrosis, this study detected the expression of miR-192-5p in tendon tissues and cells and examined whether it has a role in apoptosis, inflammation, and fibrosis of tendon cells to provide new ideas for the subsequent clinical treatment.

## 2. Material and Methods

The experimental scheme was implemented by Helsinki Declaration and approved by the Committee of People's Hospital of Ningxia Hui Autonomous Region (2020-ZDYF-028).

### 2.1. Cell Culture

Tendon cells were isolated from Achilles tendon of Sprague-Dawley rats (male, 6~8 weeks, Shanghai Slack Laboratory Animal Center) and established in an external culture. Firstly, the scabbard, blood vessels, and other tissues of the Achilles tendon were removed. The Achilles tendon tissues were then minced (1 mm × 1 mm) and digested in 3 mg/mL type I collagenase (Sigma) and 4 mg/mL neutral protease for 1 h at 37 °C. Digested cells were seeded in DMEM/F12 medium and incubated with 10% fetal bovine serum and 1% penicillin-streptomycin and incubated at 37 °C in a 5% CO_2_ incubator. The medium was changed every 3 d. Matrix colony formation of cells was observed on the 8th to 10th day of culture. P2~P3 generation cells were used for related experiments. The morphology of tendon cells was observed by microscopy and identified by collagen type I (COLI) staining.

### 2.2. Immunohistochemical Staining

Cell slides were quickly placed in cold acetone for 30 min. After soaking in the permeabilizing solution for 5 min, wash with distilled water. 50 *μ*L of 1 : 20 diluted goat serum was added dropwise and incubated at 37 °C for 15 min. After aspirating the serum, 1 : 200 dilution of COLI (ab254113, Abcam, USA) antibody was added and incubated overnight at 4 °C. After washing with PBS on a shaker, IgG H&L (HRP) secondary antibody (ab205718) was added dropwise and incubated at 37 °C for 40 min. DAB (25 mg/ml) was used for color developed and then washed with tap water. Cell slides were dehydrated with graded alcohol (80% for 2 min, 95% for 2 min, and 100% for 5 min × 2). After transparent treatment with xylene, the slides were sealed with neutral gum and observed under a microscope (× 400).

### 2.3. Cell Transfection and Treatments

NC/miR-192-5p mimic, NC/miR-192-5p inhibitor, pcDNA, and pcDNA-nuclear factor of activated T cells 5 (NFAT5) were synthesized by Invitrogen (Shanghai, China). Cells were transfected with Lipofectamine 2000 transfection reagent (Invitrogen, Shanghai, China) according to the instructions. The cells were treated with 1 ng/ml TGF-*β*1 for 0, 12, 24, 36 and 48 h after transfection for 24 h.

### 2.4. Apoptosis by Flow Cytometry

Tendon cells were harvested after 48 h of TGF-*β*1 treatment. 400 ul of 1 × binding buffer was added to 1 × 10^5^ cells in a volume of 1 ml. Then, 5 ul Annexin V-FITC was added and incubated at 25 °C for 15 min, and 5 ul PI was added to detect the percentage of apoptosis by flow cytometry. Apoptosis of tendon cells was detected by flow cytometer (BD Biosciences, COULTER-XL.MCL, NJ, USA) with EXPO32.

### 2.5. Double-Luciferase Reporter Assay

Based on the instructions of the Dual-Luciferase® Reporter Assay System kit (Promega, Beijing, China), the 3′-UTR target sequences of miR-192-5p and NFAT5 were inserted into the downstream of the luciferase gene. The expression vector and verification vector were co-transfected into tendon cells, respectively. After cell culture for 8 h, 0.5 mL of FBS containing 10% and normal DMEM medium without antibiotics were replaced and incubated in a 5% CO_2_ incubator at 37 °C for 48 h to collect cells. The fluorescence values of firefly and renilla luciferase were detected by the automatic microplate reader, and the fluorescence value of the renilla luciferase was used as an internal reference.

### 2.6. Real-Time Quantitative Polymerase Chain Reaction (RT-qPCR)

Total RNA was extracted from the samples using Trizol (Invitrogen, Shanghai, China) according to the manufacturer's instructions. The total RNA obtained was reverse transcribed into cDNA with the Reverse Transcription Kit (Qiagen, Beijing, China). A real-time PCR system (Applied Biosystems 7500, USA) was used for real-time PCR amplification. The PCR conditions were 95 °C for 1 min, 60 °C for 1 min, 72 °C for 1 min, 25-30 cycles, and 72 °C for 10 min. Relative expression was calculated by the 2^−*ΔΔ*CT^ method. U6 is the internal reference for miRNA. GAPDH is the internal reference for mRNA. Primer sequences are shown in Table 1.

### 2.7. Western Blotting

We extracted the total protein by RIPA lysate. Then, we separated 30 *μ*g protein on 10% protein electrophoresis gel and then transferred it to the PVDF membrane (Invitrogen). The PVDF membrane was blocked with 5% skim milk powder for 1-2 h, and then anti-collagen III (COLIII) (1 : 1000, Abcam, ab184993), anti-*α* smooth muscle actin (*α*-SMA) (1 : 500, Abcam, ab5694), anti- matrix metalloproteinase (MMP)-1 (1 : 1000, Abcam, ab52631), anti-MMP-8 (1 : 1000, Abcam, ab81286), anti-NFAT5 (1 : 1000, Abcam, ab3446), antitumor necrosis factor-*α* (TNF-*α*) (1 : 1000, Abcam, MA5-23720), interleukin (IL)-6 (1 : 500, Abcam, M620), anti-IL-1*β* (1 : 500, Abcam, M421B), and anti-*β*-actin (1 : 1000, Abcam, ab6276) were added and incubated overnight 4 °C. The next day, the PVDF membranes were incubated in HRP anti-mouse IgG for IP (1: 1000, Abcam, ab131368) at 25 °C for an h. The bands were detected using an exposure meter (Bio-Rad, USA) with hypersensitive chemiluminescence (HRP) detection kit (LMAI Bio, Shanghai, China).

### 2.8. Statistical Analysis

All data from at least 3 independent trials were expressed as mean ± standard deviation (SD). Comparisons between two groups were made by *t*-test, and comparisons between multiple groups were made by ANOVA test. All experimental data were subjected to three independent experiments. SPSS 13.0 was used to perform all statistical analyses. *P* < 0.05 was considered significant.

## 3. Result

### 3.1. .MiR-192-5p Was Downregulated While NFAT5 Was Upregulated in TGF-*β*1-Stimulated Tendon Cells

Firstly, tendon cells were identified by COLI staining and morphological observation. As showed in Figure 1(a), tendon cells expressed a large amount of COLI protein and were spindle-shaped. We detected the expressions of miR-192-5p and NFAT5 in tendon cells treated with TGF-*β*1 (1 ng/ml) for different times. As shown in Figure 1(b), miR-192-5p level was gradually decreased in tendon cells with the prolong of TGF-*β*1 treatment, and this was in a time-dependent manner (*P* < 0.001). Meanwhile, a gradual increasing trend was found in NFAT5 expression at both mRNA and protein levels with the increase of TGF-*β*1 administration time (Figures 1(c), 1(d), and 1(e), *P* < 0.001). The above results suggested that TGF-*β*1 stimulation is able to decrease miR-192-5p expression while increase NFAT5 expression in tendon cells.

### 3.2. MiR-192-5p Inhibits the Fibrosis in TGF-*β*1-Stimulated Tendon Cells

To verify the above speculation, we then detected the effect of miR-192-5p on the fibrosis in TGF-*β*1-treated tendon cells.  Figure 2(a) showed the expression level of miR-192-5p in the miR-192-5p mimic group was much higher than that in the NC mimic group (*P* < 0.05), suggesting the successful transfection of miR-192-5p mimic in tendon cells. Subsequently, we detected the COLIII and *α*-SMA expression in tendon cells and found that COLIII (*P* < 0.05) and *α*-SMA (*P* < 0.01) were significantly upregulated in the TGF-*β*1 group compared with the control group, while miR-192-5p mimic transfection effectively weakens this increase trend caused by TGF-*β*1 (Figures 2(b) and 2(c), *P* < 0.05). Also, we found the TGF-*β*1 stimulation resulted in an obvious elevation of MMP-1 (*P* < 0.001) and MMP-8 (*P* < 0.001), *P* < 0.01 expression, and miR-192-5p mimic transfection reversed this trend (Figures 2(d) and 2(e); *P* < 0.05 and *P* < 0.001). Together, these findings revealed that miR-192-5p inhibited the fibrosis caused by TGF-*β*1 in tendon cells.

### 3.3. .MiR-192-5p Alleviates Inflammation and Apoptosis in TGF-*β*1-Stimulated Tendon Cells

Further, we explored the effect of miR-192-5p on TGF-*β*1-caused inflammatory response and apoptosis in tendon cells. Figures 3(a) and 3(b) showed that the protein expression of TNF-*α* (*P* < 0.001), IL-6 (P < 0.001), and IL-1*β* (*P* < 0.001) in the TGF-*β*1 group was higher than the control group, while miR-192-5p partly recovered such increase (*P* < 0.01 and *P* < 0.001). Also, the percentages of cell apoptosis were detected by flow cytometry using Annexin V-FITC/PI staining. We found that TGF-*β*1 administration induced a remarkable tendon cell apoptosis (*P* < 0.001); however, the transfection of miR-192-5p mimic inhibited TGF-*β*1-induced apoptosis to some extent (*P* < 0.01, Figures 3(c) and 3(d)). Therefore, these results suggested that miR-192-5p can alleviate TGF-*β*1-induced inflammatory response and reduce apoptosis in tendon cells.

### 3.4. NFAT5 Is a Direct Target of miR-192-5p in Tendon Cells

To further understand the potential mechanism of miR-192-5p in regulating TGF-*β*1-stimulated tendon cells, we used TargetScan 7.2 (http://www.targetscan.org/vert_72) to predict the direct target of miR-192-5p and found that there was a binding site between miR-192-5p and NFAT5, as shown in Figure 4(a). In the following, we verified this result through the dual-luciferase reporter experiment and found that miR-192-5p mimic obviously reduced luciferase activity in tendon cells transfected with a reporter plasmid containing NFAT5 wild-type 3′-UTR sequence, with a statistically significant difference compared with negative control miR-192-5p mimic (*P* < 0.001), as shown in Figure 4(b). Besides, NFAT5 expression in the miR-192-5p mimic group was obviously lower than that in NC mimic group at both transcriptional and translational levels, while the miR-192-5p inhibitor was opposite (Figures 4(c), 4(d), and 4(e); *P* < 0.05 and *P* < 0.01). The above results show that NFAT5 is a direct target of miR-192-5p and is likely to be participated in miR-192-5p-mediated fibrosis and inflammatory response of tendon cells.

### 3.5. Upregulation of NFAT5 Reverses the Effect of miR-192-5p on the Fibrosis and Inflammation in TGF-*β*1-Stimulated Tendon Cells

To verify how NFAT5 involving in the regulation of fibrosis and inflammation of tendon cells, we measured the levels of COLIII and *α*-SMA proteins based on the rescue experiment. Compared with the TGF-*β*1 + miR-192-5p mimic+pcDNA group, the expressions of COLIII and *α*-SMA in the pcDNA NFAT5 transfected tendon cells were significantly increased (*P* < 0.05 and *P* < 0.01), as shown in Figures 5(a), 5(b), and 5(c). Flow cytometry results showed that the apoptosis rate of pcDNA NFAT5 transfected tendon cells was higher than that of the miR-192-5p mimic group (Figures 5(c) and 5(d), *P* < 0.01). Similarly, the expression levels of TNF-*α*, IL-6, and MMP-1 also showed the same results (*P* < 0.05, *P* < 0.01, and *P* < 0.001), as in Figures 5(e) and 5(f). These results suggest that upregulation of NFAT5 expression can reverse the effects of miR-192-5p on the fibrotic activity and inflammatory response of TGF-*β*1-stimulated tendon cells.

## 4. Discussion

Transforming growth factor (TGF)-*β* is considered to be responsible for the formation of scars such as adhesions around the healing digital flexor tendons [21]. TGF-*β*1 can accelerate wound healing, but uncontrollably can lead to pathological fibrosis and excessive collagen deposition disorder [22]. MicroRNAs are a family of small non-coding RNA molecules [23, 24], which play an important role in several human diseases, including the treatment and diagnosis of tumors [23, 25] and the musculoskeletal system [24]. Dubin et al. found that many miRNAs are involved in tendon cell development and differentiation, tendon tissue repair, and tendon cell senescence [26]. Subsequently, Xiao et al. found that miR-29a can serve as a potential therapeutic target in treating tendinopathy [27]. HumSC-EXOS may inhibit tendon adhesion by targeting miR-21a-3p by regulating p65 activity [28]. Tang et al. showed that miR-192-5p could enhance neural function by targeting FbIn2 to inhibit the activation of the TGF-*β*1 signaling pathway [29]. In this study, we found that with the increase of TGF-*β*1 treatment time, the expression level of Mir-92-5p in tendon cells gradually decreased, while the expression level of NFAT5 gradually increased. Similar to the above results, Mir-192-5p still played a role in tendon cells stimulated by TGF-*β*1. Based on the above evidence, we speculated that miR-192-5p may also play a role in TGF-*β*1-induced inflammation and fibrosis in tendon cells. However, the underlying molecular mechanisms are unclear.

Based on the above speculation, this study examined various indicators of tendon cell fibrosis and found that miR-192-5p could effectively attenuate the expression of COLIII and *α*-SMA in TGF-*β*1-stimulated tendon cells. Overexpression of *α*-smooth muscle actin (*α*-SMA) in the stroma and the inability of tendon cells to effectively transform a temporary type III collagen-rich matrix into a highly cross-linked type I collagen matrix of the original tendon promotes the accumulation of extracellular matrix [30–32]. These are all features of tendon fibrosis. Subsequently, this study also found that miR-192-5p similarly reduced the expression of MMP-1 and MMP-8 in TGF-*β*1-stimulated tendon cells. Matrix metalloproteases (MMPs) have key roles in fibrosis [33]. For example, MMP-1, MMP-8, and MMP-13 can cleave collagen molecules outside the cell matrix. These indicate that miR-192-5p inhibited TGF-*β*1-induced fibrosis in tendon cells. Similar results have been found in other studies. Studies have shown that miR-192-5p may be one of the potential biomarkers of diffuse myocardial fibrosis in patients with hypertrophic cardiomyopathy [34]. It has been shown that miR-192 can target EGR1 to prevent tubulointerstitial fibrosis in diabetic nephropathy [35]. Besides, through a systematic review and bioinformatics analysis of the relevant literature, Assmann et al. found that six miRNAs, namely, miR-21-5p, miR-29a-3p, miR-126-3p, miR-192-5p, miR-214-3p, and miR-342-3p, are involved in pathways concerning the pathogenesis of DKD, such as apoptosis, fibrosis, and accumulation of extracellular matrix, in patients with diabetic nephropathy (DKD) [36]. Meanwhile, other studies have shown that miR-192-5-p is highly expressed in adipose mesenchymal stem cell exosomes, thereby improving hyperplastic scar fibrosis [37]. In this study, Mir-192-5p not only inhibited the overexpression of *α*-SMA, but also reduced the accumulation of COLIII, thus alleviating the accumulation of extracellular matrix, and thus alleviating tendon cells fibrosis. The decreased expression of MMP-1 and MMP-8 also indicated the reduction of tendon cell fibrosis. All these results suggest that miR-192-5p regulates fibrosis not only in kidney disease but also in tendon cells.

Then, this study continued to detect the expression of inflammatory factors in each group. In this study, miR-192-5p decreased the expression of TNF-*α*, IL-6, and IL-1*β*. MiR-192-5p can alleviate the inflammatory response caused by TGF-*β*1 in tendon cells. Many studies have also found that tendon fibrosis is related to the regulation of inflammatory cytokines. Studies have shown that hepatocellular-derived exosome miR-194-5p can regulate the Rictor/Akt/FoxO1 signaling pathway, thus playing a major role in the progression of non-alcoholic fatty liver disease [38]. Hu et al. found that the upregulation of miR-192-5p in pancreatic acinar cells can reduce the inflammatory response [39]. MiR-192-5p can reduce the inflammatory response in both the liver and pancreas. Subsequently, Lou et al. found that miR-192-5p reduced inflammatory response in asthmatic mice [40]. These results are similar to the results of this study. This indicates that miR-192-5p can not only play a role in the inflammatory response of other diseases but also alleviate the inflammatory response of tendon cells caused by TGF-*β*1. The evidence is also similar to the conjecture that fibrosis is incongruous and results from persistent inflammation [41]. This study continued to detect the apoptosis of cells in each group, and the results showed that miR-192-5p could inhibit the apoptosis of tendon cells induced by TGF-*β*1. It has been shown that miR-192-5p can target FABP3 and thereby induce apoptosis in H9c2 cardiomyocytes [17]. Zhou et al. showed that miR-192-5p expression inhibited apoptosis in myeloma cells [42]. Tendon fibrosis is required to help TGF-*β*1-stimulated tendon cells return to normal function, not only in extracellular matrix degradation but also to prevent disruption of apoptotic levels. In this study, it was found that inflammatory cytokines were weakened under the action of miR-192-5p. Meanwhile, miR-192-5p inhibited TGF-*β*1-stimulated apoptosis of tendon cells. Combined with the effects of miR-192-5p in other studies, miR-192-5p can slow down the inflammatory response of tendon cells stimulated by TGF-*β*1 and inhibit apoptosis.

By prediction and validation, this study found that miR-192-5p targets binding to NFAT5. Activated T nuclear factor 5 (NFAT5), a member of the recently described Rel family of transcription factors, plays a central role in gene expression that induces immune responses [43]. This study then examined fibrosis-related and inflammatory cytokines in each group of cells and found that upregulation of NFAT5 expression increased the expression of fibrosis-related cytokines, and inflammatory cytokine expression was similarly increased. It has been shown that NFAT5 activation leads to the regulation of various genes, including some that promote inflammation [44]. Some studies have found that chronic arthritis can be treated by inhibiting the NFAT5 gene by oral administration of KRN2 and KRN5 [45]. The above studies have shown that NFAT5 has the role of promoting inflammatory response, and our study also has the same role. MiR-192-5p ameliorated the TGF-*β*1-mediated inflammatory response in tendon cells, whereas NFAT5 reversed this effect. This is also the same as the above study; by inhibiting the NFAT5 gene, the inflammatory response can be effectively improved. Besides, NFAT5 abnormalities may be responsible for the permanent fibrosis of Duchenne muscular dystrophy fibroblasts [46]. Similar to the study, our study also found that NAFT also played the same role in reversing miR-192-5p in tendon fibrosis. In terms of miR-192-5p inhibition of apoptosis, NFAT5 was able to reverse it as well. This is similar to the results of Xie et al. who showed that NFAT5 overexpression induced apoptosis in human umbilical vein endothelial cells [47]. Based on this evidence, NFAT5 reverses the effects of miR-192-5p on TGF-*β*1-mediated fibrosis and inflammatory responses in tendon cells.

## 5. Conclusion

In conclusion, miR-192-5p was expressed and downregulated in tendon cells, and the expression level gradually decreased with the prolong of TGF-*β*1 treatment. The expression of NFAT5 increased with the treatment time of TGF-*β*1. By directly targeting NFAT5, miR-192-5p inhibited TGF-*β*1-induced tendon cell fibrosis, alleviated TGF-*β*1-induced tendon cell inflammation, and reduced tendon cell apoptosis. The upregulation of NFAT5 expression reversed the effect of miR-192-5p on the fibrotic activity and inflammatory response of TGF-*β*1-stimulated tendon cells. All the above results contribute to the further understanding of the potential molecular mechanism of miR-192-5p slowing down of tendon adhesion, which is conducive to the subsequent new treatment methods and drugs.

## Figures and Tables

**Figure 1:** MiR-192-5p was downregulated while NFAT5 was upregulated in TGF-*β*1-stimulated tendon cells. (a) Immunohistochemical staining was used to detect COLI to identify tendon cells (× 400). (b) The expression of miR-192-5p in tendon cells treated with TGF-*β*1 at different times detected by RT-qPCR. (c) The mRNA expression of NFAT5 in tendon cells treated with TGF-*β*1 at different times detected by RT-qPCR. (d) The protein expression of NFAT5 in tendon cells treated with TGF-*β*1 at different times detected by Western blot.(e) Quantitative analysis of Western blot data referring to the NFAT5 protein expression. ∗∗∗*P* < 0.001 vs control.

**Figure 2:** MiR-192-5p inhibits the fibrosis in TGF-*β*1-stimulated tendon cells. (a) The expression of miR-192-5p in tendon cells transfected with NC mimic or miR-192-5p mimic detected by RT-qPCR. (b) Quantitative analysis of Western blot data referring to the protein expression of COLIII and *α*-SMA. (c) The protein expression of COLIII and *α*-SMA in tendon cells with different treatments detected by Western blot. (d) Quantitative analysis of Western blot data referring to the protein expression of MMP-1and MMP-8. (e) The protein expressions of MMP-1 and MMP-8 in tendon cells with different treatments detected by Western blot. ∗*P* < 0.05, ∗∗*P* < 0.01, ∗∗∗*P* < 0.01 vs NC mimic or control; ^#^*P* < 0.05, ^###^*P* < 0.001 vs TGF-*β*1 + NC mimic.

**Figure 3:** MiR-192-5p alleviates inflammation and apoptosis in TGF-*β*1-stimulated tendon cells. (a) The protein expression of TNF-*α*, IL-6, and IL-1*β* in tendon cells with different treatments detected by Western blot. (b) Quantitative analysis of Western blot data referring to the protein expression of TNF-*α*, IL-6, and IL-1*β*. (c) The apoptosis extent in tendon cells with different treatments detected by flow cytometry assay. (d) Quantitative analysis of flow cytometry assay data. ∗*P* < 0.05, ∗∗*P* < 0.01, ∗∗∗*P* < 0.001 vs NC mimic; ^#^*P* < 0.05, ^##^*P* < 0.01, ^###^*P* < 0.001 vs TGF-*β*1 + NC mimic.

**Figure 4:** NFAT5 is a direct target of miR-192-5p in tendon cells. (a) The predicted target binding site for miR-299-3p in the 3′UTR of NFAT5 based on the TargetScan software (http://www.targetscan.org/vert_72/). (b) Dual luciferase reporter assay results show the luciferase activity in tendon cells cotransfected with plasmid containing wild-type (WT) or mutant (MT) NFAT5 3′-UTR and miR-192-5p. (c) The mRNA expression of NFAT5 in tendon cells with different treatments detected by RT-qPCR. (d) The protein expression of NFAT5 in tendon cells with different treatments detected by Western blot. (e) Quantitative analysis of Western blot data referring to the protein expression of NFAT5. ∗*P* < 0.05, ∗∗*P* < 0.01, ∗∗∗*P* < 0.001 vs NC mimic; ^#^*P* < 0.05, ^##^*P* < 0.01, ^###^ *P* < 0.001 vs miR-192-5p mimic.

**Figure 5:** Upregulation of NFAT5 reverses the effect of miR-192-5p on the fibrosis and inflammation in TGF-*β*1-stimulated tendon cells. (a) The protein expression of COLIII and *α*-SMA in tendon cells with different treatments detected by Western blot. (b) Quantitative analysis of Western blot data referring to the protein expression of COLIII and *α*-SMA. (c) The apoptosis extent in tendon cells with different treatments detected by flow cytometry assay. (d) Quantitative analysis of flow cytometry assay data. (e) The protein expression of TNF-*α*, IL-6, and MMP-1 in tendon cells with different treatments detected by Western blot. (f) Quantitative analysis of Western blot data referring to the protein expression of COLIII and *α*-SMA. ∗*P* < 0.05, ∗∗*P* < 0.01, ∗∗∗*P* < 0.001 vs TGF-*β*1 + miR-192-5p + pcDNA.

**Table 1:** Primer sequences.

miR-192-5p	Forward: CUG-ACC-UAU-GAA-UUG-ACA-GCC
	Reverse: GGC-TGT-CAA-TTC-ATA-GGT-CAG
COLIII	Forward: TAA-AGG-GTG-AAC-GGG-GCA-GT
	Reverse: ACG-TTC-CCC-ATT-ATG-GCC-AC
*α*-SMA	Forward: GAC-AAT-GGC-TCT-GGG-CTC-TGT-AA
	Reverse: CTG-TGC-TTC-GTC-ACC-CAC-GTA
MMP-1	Forward: CTT-TGG-CTT-CCC-TAG-CAG-TG
	Reverse: TCG-CCT-TTT-TGG-AAA-ACA-TC
MMP-8	Forward: GCC-CGA-CTC-TGG-TGA-TTT
	Reverse: TGA-TGT-CTG-CTT-CTC-CCT
NFAT5	Forward: GGG-TCA-AAC-GAC-GAG-ATT
	Reverse: CAG-AGT-CGT-TGC-CCA-CA
GAPDH	Forward: CAC-TGA-GCA-TCT-CCC-TCA-CAA
	Reverse: TGG-TAT-TCG-AGA-GAA-GGG-AGG
U6	Forward: CTC-GCT-TCG-GCA-GCA-CA
	Reverse: AAC-GCT-TCA-CGA-ATT-TGC-GT

## Data Availability

The data used to support the findings of this study are available from the corresponding author upon request.
